The article "Being 40 or younger is an independent risk factor for relapse in operable breast cancer patients: The Saudi Arabia experience" was published in 2007. Journal: BMC Cancer.

# Being 40 or younger is an independent risk factor for relapse in operable  breast cancer patients: The Saudi Arabia experience

**DOI:** 10.1186/1471-2407-7-222

**Published:** 2007-12-05

**Authors:** Naser Elkum, Said Dermime, Dahish Ajarim, Ali Al-Zahrani, Adher Alsayed, Asma Tulbah, Osama Al Malik, Mohamed Alshabanah, Adnan Ezzat, Taher Al-Tweigeri

**Affiliations:** 1 Department of Biostatistics, Epidemiology, and Scientific Computing, King Faisal Specialist Hospital and Research Center, PO Box 3354, Riyadh 11211, Saudi Arabia; 2 Tumor Immunology Section, King Faisal Specialist Hospital and Research Center, PO Box 3354, Riyadh 11211, Saudi Arabia; 3 Department of Oncology, King Faisal Specialist Hospital and Research Center, PO Box 3354, Riyadh 11211, Saudi Arabia; 4 Department of Pathology, King Faisal Specialist Hospital and Research Center, PO Box 3354, Riyadh 11211, Saudi Arabia; 5 Department of Surgery, King Faisal Specialist Hospital and Research Center, PO Box 3354, Riyadh 11211, Saudi Arabia

## Abstract

**Background:**

Breast cancer in young Saudi women is a crucial problem. According to the 2002 annual report of Saudi National Cancer Registry, breast cancers that developed before the age of 40 comprise 26.4% of all female breast cancers comparing to 6.5% in the USA. Breast cancer in young patients is often associated with a poorer prognosis, but there has been a scarcity of published data in the Middle East population.

**Methods:**

Total of 867 breast cancer patients seen at King Faisal Specialist Hospital & Research Centre (KFSH&RC) between 1986 and 2002 were reviewed. Patients were divided in two age groups: ≤ 40 years and above 40 years. The clinicopathological characteristics and treatment outcomes were compared between younger and older age groups.

**Results:**

Median age at presentation was 45 years. A total of 288 (33.2%) patients were aged ≤ 40 years. Hormone receptors were positive in 69% of patients 40 and 78.2% of patients above 40 (p = 0.009). There was a significantly higher incidence of grade III tumor in younger patients compared to older patients (p = 0.0006). Stage, tumor size, lymphatic/vascular invasion, number of nodes and axillary lymph node status, did not differ significantly between the two age groups. Younger patients had a greater probability of recurrence at all time periods (p = 0.035). Young age had a negative impact on survival of patients with positive axillary lymph nodes (p = 0.030) but not on survival of patients with negative lymph nodes (p = 0.695). Stage, tumor size, nodal status and hormonal receptors had negative impact on survival. Adjuvant chemotherapy was administered to 87.9% of younger and 65.6% of older patients (*p *< 0.0001). In terms of hormone therapy, the proportion of tamoxifen treated patients was significantly lower in young age group (*p *< 0.0001). No significant difference in radiation therapy between the two groups.

**Conclusion:**

Young age (≤ 40) is an independent risk factor for relapse in operable Saudi breast cancer patients. The fundamental biology of young age breast cancer patients needs to be elucidated.

## Background

In Western societies, breast cancer is the most common cancer among women and is the leading cause of cancer mortality [1]. Breast cancer is at the top among all the malignancies seen in Saudi females, comprising of 21.8% [2]. In addition, breast cancer in young Saudi's women is a crucial problem, with the proportion of young age-onset breast cancer much higher than in western countries. According to the 2002 annual report of Saudi national cancer registry, breast cancers that developed before the age 40 accounted for 26.4% of all female breast cancers compared with only 6.5% in USA [2].

Studies have shown that the young age at diagnosis of breast cancer is associated with a poorer prognosis [3-9] or no impact on prognosis [10-15] than older age at diagnosis. Various explanations have been given to these conflicting results, including small numbers of patients, differences in patient selection criteria and inconsistent age categories used in the analyses. Indeed, it has been reported that breast carcinoma in younger patients comprises substantial clinical problems. Invasive breast carcinoma occurring in young women (defined as ages 35–40 years or younger) generally has a higher proportion of pathological features associated with more aggressive disease (Higher proportion of late stage, positive nodes, high grade, extensive intraductal component, presence of lymphatic/vascular invasion, absence of estrogen receptor, amplification or over expression of Her2/neu gene, higher S-phase fraction) compared to breast carcinoma occurring in older patients [9,16-21]. There is a paucity of published literature on experiences of treating breast cancer in a young Middle East population. To this end, it is important for clinicians to clarify the existing controversy as to whether aggressive treatment for young women with breast cancer is justified.

The aim of this study is to analyze the clinicopathological characteristics and compare the outcomes of younger breast cancer patients, to the older counterparts.

## Methods

### Patients

The pathology data and cancer registry records of the King Faisal Specialist Hospital and Research Center (KFSH&RC) from 1986 to 2002 were reviewed. KFSH&RC is a tertiary care facility and serves as the main referring center for the whole Kingdom of Saudi Arabia (KSA). Therefore, it is conceivable that the cancer pattern seen at KFSH&RC is a reflection to that seen in the whole country. This study was approved by the Research Advisory Council (Institutional Review Board) of KFSH&RC with RAC # 204006.

Only patients with stage I-III who had definitive surgery were included. Patients with distant metastasis detected at the time of diagnosis or within 4 months of surgery were excluded. Patients whose surgical margins were positive for invasive carcinoma or ductal carcinoma in situ were also excluded. Patient's records were reviewed for the following: age, tumor size, histological grade (SBR: Scarff-Bloom-Richardson classification), axillary lymph node status, presence or absence of lymphatic/vascular invasion, type of surgery and adjuvant therapy given. Estrogen receptor (ER) and progesterone receptor (PR) were determined in over 78% of cases. Disease was staged according to the American Joint Committee of Cancer (AJCC) system [22]. Disease Free Survival (DFS) was calculated as the time between diagnosis and confirmation of disease recurrence.

### Statistical analysis

Comparison of categories within a given characteristic was carried out with the Person χ^2^-test and, if any of the expected frequencies was less than five, the Fisher's exact test was used. The disease-free survival was the time between diagnosis and confirmation of disease recurrence and/or death which ever comes first. Survival analysis was conducted using Kaplan-Meier method [23], with Wilcoxon test for statistical significance. Multivariate analyses were carried out using Cox's proportional hazards model [24]. Two-sided *P*-value of < 0.05 was considered statistically significant. All statistical analyses were performed using SAS (version 9.1).

## Results

A total of 867 patients were eligible for this study, of which 288 (33.2%) were aged ≤ 40 at the time of diagnosis, and 66.8% are pre-menopausal. The median age of the patients was 45 years (range 14 – 90 years). The median tumor size was 3.0 cm (range 1 – 29.0 cm). The histology data showed that the distribution of invasive ductal carcinoma, compared to lobular carcinoma, was significantly higher in the younger age group compared to older age group (*p *= 0.0009). There was a higher proportion of double negative ER/PR status in the younger age group (*p *= 0.0086). In addition, there was a significant difference in the grade between the two groups; Grade III tumors constituted 48.5% and 36.4% of cases for patients ≤ 40 and > 40 years of age respectively. Axillary lymph node status, the most prominent prognostic factor in breast cancer, was not significantly different between the two groups. In addition, neither the tumor size, stage, lymph-lymphatic/vascular invasion nor numbers of nodes were different between the two groups. The clinicopathological characteristics of the patients in the two age groups are shown in Table 1.

**Table 1:** Clinical and pathological characteristics of all patients grouped as 40 years and > 40 years old

**Characteristics**	**Age (years)**		***P*-value**	***Total (unknown)***
	
	≤ 40 n (%)	> 40 n (%)		
Node Status				838
Positive	159 (57.8)	320 (56.8)	0.7878	(29)
Negative	116 (42.2)	243 (43.2)		
Tumor Size				824
≤ 2	93 (32.3)	186 (32.1)		(43)
3 – 5	155 (53.8))	320 (55.3)	0.8532	
≤ 5	40 (13.9)	73 (12.6)		
Number of Nodes				824
0	116 (42.3)	241 (43.1)		(43)
1 – 3	83 (30.3)	178 (31.8)	0.6731	
4 – 10	51 (18.6)	104 (18.6)		
> 10	24 (8.8)	36 (6.4)		
Stage				762
I	38 (15.0)	67 (13.1)		(105)
II	170 (67.5)	347 (68.1)	0.7259	
III	44 (17.5)	96 (18.8)		
Grade				793
I	7 (2.6)	38 (7.2)		(74)
II	130 (48.9)	297 (56.4)	0.0006	
III	129 (48.5)	192 (36.4)		
Histopathology				854
				(13)
Infiltrating ductal	270 (98.5)	520 (93.2)	0.0009	
Infiltrating lobular	4 (1.5)	38 (6.8)		
Lymph-Vascular Invasion				702
Both Positive	84 (36.7)	159 (33.8)	0.4459	(165)
Both Negative	145 (63.3)	312 (66.2)		
Hormonal Receptor Status				677
ER+ PR+	99 (44.6)	252 (55.4)	0.0086	(190)
ER- PR-	69 (31.1)	99 (21.8)		
ER+ PR-	13 (5.9)	39 (8.6)		
ER- PR+	41 (18.5)	65 (14.3)		

Table 2 shows the data obtained for the different therapeutic treatments of the 2 age groups. The proportion of breast-conserving surgery compared to mastectomy was significantly different between the two age groups (*p *= 0.0006). Adjuvant chemotherapy was administered to 87.9% of younger and 65.6% of older patients (*p *< 0.0001). In terms of hormone therapy, the proportion of tamoxifen treated patients was significantly lower in young age group (*p *< 0.0001). Adjuvant radiation therapy was administered to patients who underwent breast-conserving surgery and after mastectomy in patients who had four or more positive lymph nodes or a tumor size > 5 cm in diameter. No significant difference in radiation therapy between the two groups.

**Figure 1:** Stratified analysis of survival of breast cancer between the two age groups (≤ 40, and above 40): Patients with operable breast cancer below the age of 40 had a worse survival than the group above age 40.

**Table 2:** Treatment characteristics

**Treatments**	**Age (years)**		***P*-value**
		
	≤ 40 n (%)	> 40	
Adjuvant Anthracycline	210 (87.9)	330 (65.6)	< 0.0001
Surgery			
• Mastectomy	148 (51.4)	367 (63.5)	0.0006
• Breast conservation	140 (48.6)	211 (36.5)	
Adjuvant radiotherapy	245 (85.1)	470 (81.2)	0.1554
Adjuvant hormonal therapy	146 (58.4)	434 (81.4)	< 0.0001

Overall, the 5- and 10-year disease-free survival (DFS) of the study population was 82% and 66%, respectively. When we stratified patients by age groups, DFS was significantly poorer for the younger group (Figure 1; *p *= 0.035). Ten-year DFS of younger patients (≤ 40 years) was 60%, compared to 70% for older patients over 40 years. Tumor size, nodal involvement, number of positive nodes, pathological stages, grade, hormonal receptor status, and lymphatic/vascular invasion were significant prognostic discriminate of DFS (Table 3).

**Table 3:** Kaplan-Meier estimates of 5-year disease-free survival in relation to tumor and patient characteristics

**Characteristics**	**Number Patients**	**5-year Survival Rate**	**95% CI**	***P*-value**
Age				0.0353
≤ 40	288	0.7740	0.7201 – 0.8279	
> 40	579	0.8346	0.8007 – 0.8685	
Node Status				
• Positive	479	0.7667	0.7240 – 0.8094	< 0.0001
• Negative	359	0.8957	0.8608 – 0.9306	
Tumor Size				
≤ 2	279	0.8534	0.8062 – 0.9006	0.0052
3 – 5	475	0.8205	0.7823 – 0.8587	
> 5	113	0.7021	0.6090 – 0.7952	
Number of Nodes				
0	357	0.8953	0.8604 – 0.9302	< 0.0001
1 – 3	261	0.8057	0.7524 – 0.8590	
4 – 10	155	0.7624	0.6850 – 0.8398	
> 10	60	0.5553	0.3969 – 0.7137	
Stage				
I	105	0.8881	0.8220 – 0.9542	0.0252
II	512	0.8307	0.7954 – 0.8660	
III	140	0.7531	0.6731 – 0.8331	
Grade				0.0109
I	45	0.9750	0.9266 – 1.0000	
II	427	0.8290	0.7890 – 0.8690	
III	321	0.7681	0.7171 – 0.8191	
Histo-pathology				
• Infiltrating ductal	780	0.8145	0.7861 – 0.8429	0.2180
• Infiltrating lobular	42	0.8682	0.7404 – 0.9960	
Lymphatic/Vascular Invasion	242	0.7458	0.6835 – 0.8081	0.0002
• Both Positive	451	0.8599	0.8232 – 0.8966	
• Both Negative				
Hormonal Receptor				
Status				
• ER+ PR+	351	0.8425	0.7960 – 0.8890	0.0069
• ER- PR-	168	0.7942	0.7266 – 0.8618	
• ER+ PR-	52	0.7866	0.6688 – 0.9044	
• ER- PR+	106	0.7113	0.6000 – 0.8226	

Stratified analysis according to axillary lymph node status was performed. In lymph node-positive patients there was a significant difference in DFS between the two age groups (Figure 2; *p *= 0.030). However, in lymph node-negative patients, DFS was not significant (*p *= 0.695).

**Figure 2:** Kaplan-Meier survival analysis of patients with positive axillary lymph nodes and effects on survival stratified by age groups ≤ 40 years, and above 40 years. Patients with positive axillary lymph nodes and young age have worst survival. (P = 0.030).

In multivariate analysis, young age (≤ 40 years) remained a significant predictor of relapse when entered into a model containing all potential demographic, pathologic and immunohistochemical variables (Table 4. Hazard Ratio (HR), 1.5; confidence interval, 1.0 – 2.2; *p *= 0.0352).

**Table 4:** Multivariate analysis for predictors of DFS based on the Cox proportional hazards regression model

**Variables**	**HR**	**95% CI**	***P*-value**	***Overall P-value***
Age				
≤ 40	1.51	1.03 – 2.23	0.0352	
> 40	1	–	–	
Node Status			< 0.0001	
Positive	2.24	1.53 – 3.29		
Negative	1	–		
Tumor Size				0.0170
≤ 2	1	–	-	
3 – 5	1.28	0.85 – 1.92	0.2440	
> 5	2.23	1.20 – 4.36	0.0118	
Stage				0.0002
I	0.55	0.35 – 0.86	0.0093	
II	0.44	0.22 – 0.87	0.0195	
III	1	--	-	
Grade				0.0078
I	1	--	--	
II	0.95	0.55 – 1.64	0.8550	
III	1.21	0.69 – 2.13	0.4978	
Lymph-Vascular Invasion				
Both Positive	1.11	0.78 – 1.58	0.5708	
Both Negative	1	--	--	
Hormonal Receptor Status				0.0027
ER+ PR+	1	--	--	
ER- PR-	1.21	0.79 – 1.83	0.3786	
ER+ PR-	1.17	0.60 – 2.29	0.6390	
ER- PR+	1.79	1.11 – 2.89	0.0179	

## Discussion

Patients included in this study illustrate interesting characteristics where 33.2% are young (≤ 40 years) and 66.8% are pre-menopausal. While the median age at presentation is around 63 years in the United States and Western Europe, the median age at presentation in this study is 45 years. The young age of patients in this study is attributed to the overall age distribution in the KSA, where 50% of the population is less than 15 years of age and only 3% are older than 65 years. These patients' characteristics are in sharp contrast with those reported in the West.

Gajdos *et al *[25] reported that patients diagnosed with breast cancer before age 36 differ from older patients in several respects. The younger age group presents more often with more advanced and aggressive cancer. In spite of aggressive treatment (mastectomy and chemotherapy) in the younger age group, local and distant failure rates are higher than for patients 36 and older. The higher rate of local recurrence in patients less than 36 years reflects an excess number of local recurrences in patients treated with breast conservation. In the present study, we have found that patients ≤ 40 years were treated more often with breast-conserving surgery compared to mastectomy (48.6% versus 36.5%, *p *= 0.0006), adjuvant chemotherapy (87.9% versus 65.6%, *p *< 0.0001), and less often with tamoxifen (*p *< 0.0001). Our current findings are in agreement with what have been reported by Gajdos *et al *investigating breast cancer in young women [25]. It is important to mention that similar protocols for the treatment of breast cancer patients were used in both USA and KSA and this may reflect the similarity of both studies.

Our results show that young age is a critical prognostic factor in women with breast cancer in Saudi Arabia. Among all studied prognostic factors, the distribution of grade, histology, and hormonal receptor status showed a significant difference between the two age groups in our patient population.

The results of the present investigation showed that being young age at diagnosis (≤ 40 years) is an independent prognostic factor for disease-free survival in addition to nodal status, pathological tumor size, stage and hormonal receptor status. We performed subgroup analysis by investigating patients with negative versus positive lymph nodes and had different results. Young age had a significant impact on survival in patients with positive lymph nodes but not in patients with negative lymph nodes.

The present findings support previous reports showing that women diagnosed with breast cancer at younger age have a poorer prognosis compared with their older counterparts [8,18,26-28]. The extensive heterogeneity of breast cancer complicates the precise assessment of tumor aggressiveness which makes therapeutic decisions difficult and treatment impropriate in some cases [28]. Therefore, it is very important to understand the interactions between the genetic complexity and the environmental factors which modulate the onset and progression of breast cancer in young women which may help in designing a personalized treatment for this patient population. For example, it has been demonstrated that about 15–30% of western breast cancer women aged less than 35 years are likely to have germ-line BRCA1 or BRCA2 mutations [29,30]. Similar results were reported for BRCA1 and BRCA2 mutations in Korean women with breast cancer at a young age (< 40 years) [31] and also for BRCA1 mutations in a series of Singaporean Chinese women with early onset (cut-off of 40 years) [32]. Study on BRCA1 and BRCA2 mutations in Saudi women older than 40 years with breast cancer concluded that mutations in these genes are likely to contribute to the pathogenesis of familial breast cancer in the Kingdom of Saudi Arabia [33]. A recent interesting tissue microarray study by Eerola *et al *[34]demonstrated that tumors of BRCA1 and BRCA2 positive-mutations aged 50 years or more (postmenopausal) differed significantly from those of younger age group (premenopausal) with similar mutations. This difference may reflect diverse biological behavior and pathways of tumor development among the older and the younger BRCA1 and BRCA2 patients, with impact also on prognosis and survival. Overall, there is an emerging picture indicating that breast cancer risk in BRCA1 and BRCA2 positive women are substantially higher than in the general population and the genes are considerably affected by non-genetic, environmental factors and by additional genetic modifiers [35]. In the light of the high incidence of breast cancer in young Saudi women [2], mutation study of these genes and gene-expression profile, which is a more powerful predictor of the outcome of disease in young patients with breast cancer [36], are extremely warranted.

## Conclusion

In conclusion, we show that operable Saudi young breast cancer patients (≤ 40 years old) have a worse prognosis than older patients. Increasing tumor size, late stage, positive lymph nodes, young age at diagnosis, and hormonal receptor status were independent prognostic indicator for survival. Indeed younger patients have a poorer disease free survival. The underlying biology of breast cancer among patients needs to be elucidated.

## List of abbreviations

KSA = Kingdom of Saudi Arabia, KFSH&RC = King Faisal Specialist Hospital & Research Centre, SEER = Surveillance, Epidemiology and End Results; SBR = Scarff-Bloom-Richardson classification; ER = Estrogen receptor; PR = progesterone receptor; DFS = disease-free survival.

## Competing interests

The author(s) declare that they have no competing interests.

## Authors' contributions

NE contributed to the database, data collection, analysis, writing and editing of the manuscript. SD helped draft, edit and revised the manuscript. DA selected cases and contributed to the database; AT carried out the pathological diagnosis; TT selected cases, reviewed medical records, and writing and editing of the manuscript. AA, AZ, OA, MA and AE conceived of the study and participated in its coordination. All authors read and approved the final manuscript.

## Pre-publication history

The pre-publication history for this paper can be accessed here:


